# Distinctive Metabolism-Associated Gene Clusters That Are Also Prognostic in Intrahepatic Cholangiocarcinoma and Hepatocellular Carcinoma

**DOI:** 10.1155/2022/6595989

**Published:** 2022-09-19

**Authors:** Linchao Ding, Shilong Ning, Weijian Hu, Yadong Xue, Shi'an Yu

**Affiliations:** ^1^Central Laboratory, Affiliated Jinhua Hospital, Zhejiang University School of Medicine, Jinhua, China; ^2^Department of Clinical Nutrition, Affiliated Jinhua Hospital, Zhejiang University School of Medicine, Jinhua, China; ^3^Department of Hepatobiliary and Pancreatic Surgery, Affiliated Jinhua Hospital, Zhejiang University School of Medicine, Jinhua, China

## Abstract

**Objective:**

To offer new prognostic evaluations by exploring potentially distinctive genetic features of hepatocellular carcinoma (HCC) and intrahepatic cholangiocarcinoma (ICC).

**Methods:**

There were 12 samples for gene expression profiling processes in this study. These included three HCC lesion samples and their matched adjacent nontumor liver tissues obtained from patients with HCC, as well as three ICC samples and their controls collected similarly. In addition to the expression matrix generated on our own, profiles of other cohorts from The Cancer Genome Atlas (TCGA) program and the Gene Expression Omnibus (GEO) were also employed in later bioinformatical analyses. Differential analyses, functional analyses, protein interaction network analyses, and gene set variation analyses were used to identify key genes. To establish the prognostic models, univariate/multivariate Cox analyses and subsequent stepwise regression were applied, with the Akaike information criterion evaluating the goodness of fitness.

**Results:**

The top three pathways enriched in HCC were all metabolism-related; they were fatty acid degradation, retinol metabolism, and arachidonic acid metabolism. In ICC, on the other hand, additional pathways related to fat digestion and absorption and cholesterol metabolism were identified. Consistent characteristics of such a metabolic landscape were observed across different cohorts. A prognostic risk score model for calculating HCC risk was constructed, consisting of *ADH4*, *ADH6*, *CYP2C9*, *CYP4F2*, and *RDH16*. This signature predicts the 3-year survival with an AUC area of 0.708 (95%CI = 0.644 to 0.772). For calculating the risk of ICC, a prognostic risk score model was built upon the expression levels of *CYP26A1*, *NAT2*, and *UGT2B10*. This signature predicts the 3-year survival with an AUC area of 0.806 (95% CI = 0.664 to 0.947).

**Conclusion:**

HCC and ICC share commonly abrupted pathways associated with the metabolism of fatty acids, retinol, arachidonic acids, and drugs, indicating similarities in their pathogenesis as primary liver cancers. On the flip side, these two types of cancer possess distinctive promising biomarkers for predicting overall survival or potential targeted therapies.

## 1. Introduction

Primary liver cancer is one of the most common malignancies worldwide with steadily increasing incidence rates globally despite the benefits gained from the control of viral infections in some regions [1, 2]. According to GLOBOCAN, 905,677 new cases of liver cancer developed in 2020, taking up 4.7% of all new cancer cases worldwide. In the same year, deaths resulting from liver cancer contributed to 8.3% of all cancer deaths. The burden that primary liver cancer has imposed on the global economy and healthcare system makes it an urgent task to understand the pathogenesis of liver cancer better. Two histological types contributed to most cases of primary liver cancer: hepatocellular carcinoma (HCC) and intrahepatic cholangiocarcinoma (ICC), which account for more than 70% and around 15%, respectively [3, 4]. Multiple established risk factors have been confirmed to be responsible for the development of HCC, such as chronic infection of hepatitis B or C virus and exposure to aflatoxin-b1 [5, 6]. However, despite advanced progress in finding associations between ICC and cirrhosis, viral infections, or metabolic disorders [7–10], most cases of ICC lack well-confirmed risk factors thus necessitating further exploration for markers of early surveillance or methods to prolong survival [11]. Clinically, the site of origin or histology of liver cancer sometimes, unfortunately, cannot be identified, and the diagnosis can be rather tricky when it comes to differentiating HCC and ICC, despite their different origins and histological features; this is especially true when extrahepatic malignancies metastasize to the liver and complexify the whole situation [4, 12]. Contrast-enhanced ultrasound on top of baseline ultrasound has been proven to improve the differential diagnostic performance [13], and novel biomarkers are being worked on to rule out metastasized adenocarcinoma and even narrow down the diagnoses to one of these two major types of primary liver cancer [12]. The fact is, even though extensive conventional histology and immunohistochemistry are supposed to be able to tell the differences between HCC samples and ICC samples, many ICC cases are found when patients are screened for high risk or presumed diagnosis of HCC. Some are even confirmed in those who are undergoing hepatic resection or transplantation due to HCC [4]. The difficulties of differential diagnoses might have contributed to some of HCC's risk factors being shared as features related to ICC. Metabolism-related factors such as obesity and diabetes have been proven to be associated with the pathogenesis of HCC or primary liver cancer in general; particular pathways involving lipid metabolism are even speculated to be promising in serving as therapeutic targets [14–17]. ICC resembles HCC more than extrahepatic biliary carcinoma in that highly presented albumin can be found in ICC, which is a highly specific and sensitive marker for HCC. It is reasonable to hypothesize that HCC and ICC share the same progenitor cells with the evidence that both types were developed when using an albumin-Cre system with liver-specific inactivation of *Nf2* and *Mst1*/*Mst2* in genetically engineered mouse models [18–21].

With samples of tumor lesions and paratumor normal samples acquired from patients confirmed with HCC and ICC, the differentiation analyses and functional analyses in this study confirmed the dysregulated metabolism-related genes in both types, yet with distinctive landscapes of metabolism changes. This was validated on a larger scale with the expression profiles available in The Cancer Genome Atlas program and the Gene Expression Omnibus. We aimed to develop a prognostic model of distinct metabolism-related genes (MRGs) for each histologic type and successfully achieved this in HCC. Another set of MRGs targeting different pathways compared to HCC was included in the model built for predicting the prognosis of ICC. Though the model itself was not satisfyingly validated across all the cohorts, these genes seemed to be consistently related to the prognosis of ICC. We hope this observation will help reveal the characteristic metabolism-related landscapes of HCC and ICC to differentiate them and also aid in predicting the prognostic status of patients with HCC and ICC.

## 2. Materials and Methods

### 2.1. Sample Collection

Three HCC lesion samples and their matched adjacent nontumor liver tissues were obtained from patients with HCC who received curative surgery at Affiliated Jinhua Hospital, Zhejiang University School of Medicine, Zhejiang Province, China. ICC samples were collected similarly. There were in total 12 samples included for gene expression profiling processes. The related clinicopathological features of the enrolled patients are presented in Supplementary Table 1. All samples were obtained with informed consent of the patients. This study complied with the standards of the 1975 Declaration of Helsinki, and the experiments were approved by the Ethics Committee of Affiliated Jinhua Hospital, Zhejiang University School of Medicine.

### 2.2. Gene Expression Profiling

#### 2.2.1. mRNA Library Constructing and Sequencing

RNA was extracted from samples, and 1 *μ*g total RNA was used for the following library preparation. The poly(A) mRNA isolation was performed using Oligo(dT) beads. The mRNA fragmentation was performed using divalent cations and high temperatures. Priming was performed using random primers. First-strand cDNA and the second-strand cDNA were synthesized. The purified double-stranded cDNA was then treated to repair both ends and add a dA-tailing in one reaction, followed by a T-A ligation to add adaptors to both ends. Size selection of adaptor-ligated DNA was then performed using DNA clean beads. Each sample was then amplified by polymerase chain reaction (PCR) using P5 and P7 primers, and the PCR products were validated. Primer sequences for P5 and P7 are shown in Supplementary Table 2. Then, libraries with different indexes were multiplexed and loaded on an Illumina HiSeq instrument for sequencing using a 2 × 150 paired-end (PE) configuration according to the manufacturer's instructions.

#### 2.2.2. Quality Control

Technical sequences including adapters, PCR primers, or fragments thereof and quality of bases lower than 20 were removed by processing the data with Cutadapt (V1.9.1, Phred cutoff: 20, error rate: 0.1, adapter overlap: 1 bp, min. length: 75, and the proportion of *N*: 0.1) to be high-quality clean data.

#### 2.2.3. Alignment

Firstly, reference genome sequences and gene model annotation files of relative species were downloaded from genome websites, such as UCSC, NCBI, and ENSEMBL. Secondly, Hisat2 (v2.0.1) was used to index the reference genome sequence. Finally, clean data were aligned to the reference genome via software Hisat2 (v2.0.1).

#### 2.2.4. Expression Analysis

In the beginning, transcripts in fasta format are converted from known gff annotation files and indexed properly. Then, with the file as a reference gene file, HTSeq (v0.6.1) estimated gene and isoform expression levels from the pair-end clean data.

### 2.3. Datasets from Online Databases

Databases such as The Cancer Genome Atlas (TCGA) program and the Gene Expression Omnibus (GEO) were searched, and the following expression datasets were selected: hepatocellular carcinoma data collection (TCGA-LIHC), matrix of samples categorized as ICC in TCGA's study of cholangiocarcinoma (TCGA-CHOL), ICC matrix including 30 samples from GSE107943, and HCC matrix of the training cohort from GSE14520. In addition, one cohort was established by randomly selecting 25 ICC cases and 25 HCC cases from TCGA-LIHC and TCGA-CHOL with complete overall survival and detailed status; then, normalization of the gene expression level was conducted through *z*-score, and batch effects were removed. A validation cohort was constructed from the aforementioned GSE datasets after similar processes.

### 2.4. Identification of Key Genes

#### 2.4.1. Differential Analyses

With the cut-off criteria set as |log_2_(foldchange)| >1 and *p* value < 0.05, we screened the differentially expressed genes (DEGs) via the “limma” R package.

#### 2.4.2. Functional Analyses

Functional analyses and annotations were conducted based on the Kyoto Encyclopedia of Genes and Genomes (KEGG) and Gene Ontology (GO) database, with the Database for Annotation, Visualization, and Integrated Discovery (DAVID). Pathways with *p* < 0.05 were considered statistically significant.

#### 2.4.3. Predicted Protein Interaction Network Analysis

With a minimum required interaction score setting of 0.4, the Search Tool for the Retrieval of Interacting Genes/Proteins (STRING, https://string-db.org/) database was employed to construct a PPI network, which depicts the interactions of proteins encoded by DEGs. The MCL clustering method was applied afterwards with an inflation parameter equal to 0.3. Significantly enriched clusters with gene numbers over 10 were selected for further analyses.

#### 2.4.4. Acquisition of the List of Metabolism-Related Genes

The list of metabolism-related genes (MRGs) was acquired similarly to Jiang et al. by extracting them from metabolic pathways annotated in the KEGG database [22].

#### 2.4.5. Gene Set Variation Analysis (GSVA)

Sets of genes encoding significantly enriched protein clusters generated from PPI analyses were used as individual signatures. The enrichment score of each signature in each sample was calculated based on published methods [23]. Receiver operating characteristic curves were conducted to evaluate the performance of each score in classifying the two histological types. The subsequent prognosis model was built on genes selected from clusters with high classifying abilities.

### 2.5. Establishment of Prognostic Models

To establish a prognostic model specifically for each histological type, first, we identified genes that were associated with prognosis with univariate Cox analyses. Genes with *p* < 0.05 were regarded as prognosis-associated metabolic genes. Among them, multivariate Cox analyses were then conducted to build the final model. After Stepwise regression analysis plus the Akaike information criterion (AIC), the optimal one was selected.

## 3. Results

### 3.1. Different Landscapes of Metabolism-Related Pathways Were Observed in HCC and ICC

We first conducted three differential analyses with our sequenced samples: (1) three HCC samples versus their matched adjacent nontumor tissue, (2) three ICC samples versus their matched adjacent nontumor tissue, and (3) three HCC samples versus 3 ICC samples. The volcano plots depicting significantly upregulated and downregulated genes are shown in Figures 1(a)–1(c) (|logFC| > 1 and *p* value < 0.01). Among all 999 DEGs identified by comparing HCC and ICC, 86 genes were also specifically differentially expressed in HCC compared to its matched nontumor tissue, while 566 DEGs were specifically differentially expressed in ICC compared to its matched nontumor tissue (Figure 1(d)).

We conducted subsequent functional analyses on the abovementioned DEGs based on the KEGG database (Figures 2(a), 2(b), 3(a), and 3(b)). As the top 20 KEGG enrichment revealed, an abundance of genes in both HCC and ICC was related to metabolic pathways, such as the metabolism of fatty acids, retinol, amino acids, and other important biological substances.

Functional analyses based on the GO database consistently revealed the abundance of metabolism-related genes, with molecular functions such as binding and catalytic activity (Figures 2(a) and 2(b)). We speculated that metabolism-related genes might have been playing important roles in the pathogeneses of HCC and ICC. From the differently enriched specific pathways exhibited by HCC and ICC in functional analyses, it was also natural to hypothesize that HCC or ICC had differently dysregulated metabolic pathways. If we were able to capture this difference, we might be able to understand better the evolvements and outcomes of these two histological types.

To further this hypothesis, we first took a glance at our 12 samples with a PCA using the expression matrix of all metabolism-related genes (Figure 3). The nontumor samples adjacent to tumor sites were not separated using this metabolic feature; however, the difference between HCC and ICC samples could be well appreciated. This evidence added up to our speculation but was limited by the number of samples we had. Thus, TCGA-CHOL and TCGA-LIHC were employed in our later analyses. Only samples with histological type and tumor site as intracellular cholangiocarcinoma were selected from TCGA-CHOL.

Similarly, differential analyses were conducted for HCC and ICC with their matched nontumor samples (Figure 4(a)), and then, we identified all 217 metabolism-related genes that were also differentially expressed in both HCC and ICC (Figure 4(b)). Consistently, we found that these metabolism-related genes were significantly associated with fatty acid metabolism (ko00071), retinol metabolism (ko00830), and drug metabolism (ko00983), as well as many other substances essential for biosynthesis (Figure 4(c)).

### 3.2. From Key Clusters to Key Genes/Signatures

We further explored the proteins coded by these 217 genes with the STRING database. A protein-to-protein network was constructed, and 43 clusters were identified from this network, with 9 of them containing more than 10 proteins (MCL clustering, with inflation parameter = 3, Table 1).

The networks of these clusters were reconstructed separately and shown in Figure 5.

Till this step, we have acquired key clusters of genes that (1) were differentially expressed between HCC and ICC versus their adjacent nontumor tissue, (2) were highly related to metabolic pathways, and (3) could be associated with the pathways validated to be altered in our samples but to different extents in HCC and ICC. To test if any of these clusters would be able to dictate the different landscapes in terms of metabolism exhibited by HCC and ICC, we started with a small cohort consisting of 25 randomly selected ICC samples from TCGA-CHOL and 25 HCC samples from TCGA-LIHC. There was a big difference in the original datasets from TCGA-CHOL and TCGA-LIHC in terms of sample size; by selecting randomly and removing batch effects, this cohort with complete clinical characteristics (age, gender, survival months, and end-event) served as the input for our next analyses to narrow down the number clusters.

GSVA was conducted using genes from 9 clusters as separate signatures. The scores were used as features distinctively to differentiate two histological types apart. The ROC curves were plotted for each one of them (Table 2) and visualized together in Figure 6(a).

When using the gene set variation scores of clusters 1 and 2 as features, HCC was differentiated from ICC very well. The combination of the two achieved an even better result with an AUC equal to 0.867 (CI: 0.762 to 0.973, Figure 6(b)), and ICC tended to score significantly higher than HCC (Figure 6(c)).

### 3.3. Prognosis-Related Genes and Signature Building or Verification

In the next step, we included all samples with complete clinical information from TCGA-LIHC and TCGA-CHOL and explored the possibility of exploiting genes from clusters 1 and 2 to build prognosis-related models that are specific to each histological type. Univariate Cox regression analyses were first performed, fourteen genes from clusters 1 and 2 were proven to be prognosis-related (*p* < 0.05) in HCC, and comparatively, three genes from clusters 1 and 2 were prognostic for ICC (Table 3). Multivariate Cox regression analyses were then performed to find the optimal models, and for 14 genes of HCC, iteration was carried out with *Step* function in R, and models with the smallest AIC value were selected.

According to the results of multivariate Cox regression analysis, we constructed a prognostic risk score model for calculating HCC risk as follows: risk score of HCC (RS_HCC) = (−0.1393 × expression value of *ADH4*) + (0.2214 × expression value of *ADH6*) + (−0.1339 × expression value of *CYP2C9*) + (0.1017 × expression value of *CYP4F2*) + (−0.0978 × expression value of *RDH16*), with AIC value =1304.0967.

We ranked the risk score of each subject and listed them along with the expression heat map and their survival status in Figure 7. As the dot plot and Kaplan-Meier curve depicted, subjects with higher RS_HCC had significantly lower survival times compared to those with lower risk scores (HR = 2.92, 95%CI = 1.98 to 4.29, *p* = 1.5e − 08). This signature predicts the 3-year survival with an AUC area of 0.708 (95%CI = 0.644 to 0.772).

Similarly, we constructed a prognostic risk score model for calculating ICC risk as follows: risk score of ICC (RS_ICC) = (−1.1988 × expression value of *CYP26A1*) + (0.1217 × expression value of *NAT2*) + (0.2819 × expression value of *UGT2B10*), with AIC value =100.3791. Likewise, the risk scores of each subject were ranked and listed along with the expression heat map of these three genes and their survival status in Figure 8. Subjects with higher RS_ICC had significantly lower survival times compared to those with lower risk scores (HR = 11.94, 95%CI = 2.63 to 54.17, *p* = 7.1e − 05). This signature predicts the 3-year survival with an AUC area of 0.806 (95%CI = 0.664 to 0.947). However, extra cautions should be noted when interpreting these considering the rather limited number of cases in this dataset in comparison to TCGA-LIHC.

### 3.4. Verification in GEO

We validated the value of applying these two models in predicting the survival of patients with primary liver cancer. Two datasets were chosen and combined with batch effect removed and expression levels standardized: one was from GSE107943 collected from patients with ICC and a subset with a similar number of patients with HCC from GSE14520. With the annotation files available, unfortunately, we failed to detect the expression of *ADH4* and *UGT2B10* from these expression matrices. They were therefore eliminated from the equation. Except that, two risk score models were both applied regardless of the original histological types. RS_HCC significantly indicated longer survival in patients with HCC (*p* = 5.4*e* − 03), and low RS_ICC in HCC patients indicated a worse prognosis (*p* = 0.04) (Figure 9(a)). Neither score model depicted any differences in survival between low-risk and high-risk patients to a statistically significant level (Figure 9(b)). Considering that one major factor (*UGT2B10*) was missing from the calculation and the remaining two (*CYP26A1*, *NAT2*) contributed to the risk score oppositely, we verified the value of using the expression levels of *CYP26A1* and *NAT2* separately in predicting the survival, in this cohort. It turned out that for this cohort, only the expression of *NAT2* truly reflected the risk score of ICC (Figures 9(c) and 9(d)).

## 4. Discussion

Two histologic types HCC and ICC take up more than 80% of all primary liver cancer cases. The latter along with a less frequent mixed type of both types has a poor prognosis compared with HCC [24, 25]. For HCC, especially nonresectable HCC, transarterial chemoembolization can achieve moderate therapeutic effects among patients at early stages, but the long-term benefits of this only treatment are not satisfying due to refractoriness and the negative effects on normal liver tissue [26, 27]. On another aspect, the existence of the combined hepatocellular cholangiocarcinoma suggested the overlap of two major histological types, but the diagnosis is primarily morphological with additional immunostaining. What is more, despite the probable common risk factors for developing HCC and ICC, the prevention plans, as well as the treatments, differ in these two types thus necessitating proper and precise classification. Research has been focused on multiple methods including multiphase computerized tomography [28], magnetic resonance imaging [29], contrast-enhanced ultrasound [13, 30], and biomarkers to differentiate HCC from ICC [12].

The liver is the main hub for the metabolism of various kinds of biological substances, especially lipids. Lipid metabolism is essential not only for the generation of energies but also for the basic cellular growth and molecular signalling in many oncogenic pathways. Complicated remodelling of important metabolic pathways such as lipid degradation has been theorized to be associated with the development of liver cancer. Upregulated lipid synthesis and inhibition of degradation supply the malignant cells with basic building materials and raw ingredient for signalling molecules to accelerate the proliferation and ensure their proper communication [31].

HCC itself, on the other hand, can influence lipid metabolism; thus, the lipid profiles or related markers may be also indicative of prognosis [32]. It is natural to consider the therapeutic value of agents specifically targeting lipid metabolism to achieve discriminative clinical benefits in liver cancer [14]. There are numerous inhibitors targeting enzymes involved in *de novo* lipogenesis that have been produced [33–35], yet further validations in animal models and advanced clinical trials are still needed. Considering the natural function of the liver and the association of malignancies developed here with metabolism, it is reasonable to hypothesize that dysregulation of metabolism-related genes (MRGs) might have been important in the pathogeneses of HCC and ICC, and HCC and ICC may possess different signatures of MRGs.

In the first part of this study, we revealed the different landscapes of metabolism-related pathways in HCC versus ICC by analyzing our sequencing data. The differentially expressed genes in each histological type in comparison to their matched nontumor samples are enriched into similar pathways related to metabolism. To narrow the genes down, we only performed functional analysis for genes that are also differentially expressed between HCC and ICC. Fatty acid degradation, retinol metabolism, and arachidonic acid metabolism turn out to be the top three pathways in HCC. In ICC, besides these same pathways, pathways related to fat digestion and absorption and cholesterol metabolism are also significantly enriched. This is following previously mentioned evidence of dysregulated lipid metabolism in liver cancer and validates the possibility of exploiting the value of lipid synthesis inhibitors in the treatment.

The dissimilarities of HCC versus ICC were depicted in the principal component analysis using the expression matrix of all metabolism-related genes. Overlap of the nontumor samples implied the resemblance of the baseline metabolic features while the clear separation of ICC and HCC samples indicated their distinctive metabolic nature. To further validate this observation on a larger scale, a similar series of differential analyses plus functional analyses were done in TCGA-LIHC and TCGA-CHOL. We eventually aimed to identify key genes that (1) are differentially expressed in both HCC and ICC compared to the nontumor samples and (2) lead to the same metabolic functions but to different extents in these two histological types. Thus, this time, the common DEGs which are also metabolism-related genes were picked for functional enrichment. Interestingly, we consistently observed significantly enriched pathways in retinol metabolism, fatty acid degradation, and arachidonic acid metabolism. Other than these, pathways involving enzymes in drug metabolism such as the cytochrome P450 system was also significantly enriched. This superfamily contains enzymes that are important for the clearance of various compounds including drugs, as well as for the synthesis and breakdown of hormones. Specific mutations of certain members within this family affect the efficacy of chemotherapeutical treatment [36], and dysregulations have been linked with the carcinogenesis of HCC and ICC [37]. The transcriptomic information of the cytochrome P450 system can provide insights into both the identification and prognosis of HCC [38].

From the DE-MRGs identified from TCGA, a complex predicted interactive network was constructed. Nine protein clusters with strong local clustering efficiency were identified. Interestingly, when we traced back to the genes that encode these clusters of proteins, we found that these gene sets varied significantly in HCC and ICC. They exhibited distinctive features in terms of most of these clusters in that the GSVA score calculated well classified these two histological types (6 out of 9 with AUC over 0.6). This further solidates the hypothesis that different landscapes of MRGs exist in HCC and ICC, even though they share some dysregulated metabolic pathways.

In HCC, five genes were included eventually in our prognostic model: *ADH4*, *ADH6*, *CYP2C9*, *CYP4F2*, and *RDH16.* All-trans-retinol dehydrogenase 4 (ADH4) catalyzes the nicotinamide adenine dinucleotide- (NAD-) dependent oxidation of either all-trans-retinol or 9-cis-retinol [39]; retinol dehydrogenase 16 (RDH16) also oxidizes the same substrates with a preference for NAD [40–42] but with higher activity toward cellular retinol-binding protein- (CRBP-) bound retinol than with free retinol [41]. Another gene associated with retinol metabolism but also a member in the CYP450 superfamily showed up in the prognostic model of ICC: *CYP26A1*. The protein it encodes is a cytochrome P450 monooxygenase involved in the metabolism of all-trans-retinoic acid (ATRA). ATRA is an important signalling molecule that binds to retinoic acid receptors and regulates gene transcription. The proper function of this enzyme tightly relies on the interaction with cytochrome P450 reductase, and it cannot metabolize certain isomers of retinoic acid such as 9-cis and 13-cis stereoisomers [43–45]. Possible therapeutic effects of ATRA in liver cancer especially HCC have been extensively researched [46–51].

There are two more genes encoding enzymes of the CYP450 family. One is *ADH6*, encoding the alcohol dehydrogenase 6, which also consumes NAD^+^. It is involved in the metabolism of various endogenous substrates, including fatty acids and steroids [52–58]. It catalyzes the epoxidation of double bonds of polyunsaturated fatty acids [53, 54, 58] and metabolizes cholesterol toward 25-hydroxycholesterol, a physiological regulator of cellular cholesterol homeostasis [52]. The last gene, CYP4F2, is involved in the metabolism of fatty acids and eicosanoids [59–64] and participates in the conversion of arachidonic acid to omega-hydroxyeicosatetraenoic acid (20-HETE) [59, 60, 62]. CYP4F2 plays a role in the oxidative inactivation of eicosanoids, including both proinflammatory and anti-inflammatory mediators [60, 62, 63, 65, 66].

In ICC, three genes were included in the prognostic model: *CYP26A1*, *NAT2*, and *UGT2B10*. As previously discussed, one of them shared a similar role in processing retinoic acid. The rest two, on the other hand, are more involved in drug/toxin metabolism. *NAT2*, for example, encodes arylamine N-acetyltransferase 2, which participates in the detoxification of a lot of hydrazine and arylamine drugs. It catalyzes the acetylation of various amine substrates and most importantly can bioactivate several known carcinogens. Meanwhile, *UGT2B10*-encoded uridine 5′-diphosphate-glucuronosyltransferase is of major importance in the conjugation and subsequent elimination of potentially toxic xenobiotics and endogenous compounds. This prognostic model was not well validated in the GEO cohort probably due to the small sample size in the original TCGA-CHOL. Comparatively, the model for HCC which was developed from a large cohort was more convincing. However, the fact that the expression of *NAT2* is consistently prognostic still provided some insights to explore the metabolic pattern distinctively for ICC.

Overall, the hypothesis is further validated that HCC and ICC share some common metabolism-related pathways especially the metabolism of fatty acids, retinol, arachidonic acids, and drugs, indicating similarities in their pathogenesis as primary liver cancers. In the meantime, they also vary when it comes to specific enzymes and regulators in the essential pathways, which implies different promising biomarkers for predicting overall survival or potential targeted therapies.

## Figures and Tables

**Figure 1:** Differentially expressed genes between HCC and normal (a), between ICC and normal (b), and between HCC and ICC (c). (d) DEGs that are differentially expressed between two histological types and significantly regulated in each type, respectively, compared to normal tissue.

**Figure 2:** Significantly enriched pathways based on KEGG and GO databases: (a) functional pathways exhibited by genes that are differentially expressed in HCC compared to its control and differentially expressed compared to ICC samples (left: summary of enriched pathways in KEGG annotation; middle: top 20 enriched pathways; right: Gene Ontology classification); (b) functional pathways exhibited by genes that are differentially expressed in ICC compared to its control and differentially expressed compared to HCC samples (left: summary of enriched pathways in KEGG annotation; middle: top 20 enriched pathways; right: Gene Ontology classification).

**Figure 3:** Principal component analysis indicated the distinctive natures of ICC and HCC versus the nontumor site in terms of metabolism-related genes.

**Figure 4:** Differential analyses conducted in TCGA-CHOL and TCGA-LIHC in comparison with nontumor samples (a) revealed 217 commonly differentiated metabolism-related genes (b) significantly enriched to fatty acid metabolism, retinol metabolism, and drug metabolism (c).

**Figure 5:** Predicted protein interaction analysis revealed 9 enriched major clusters of proteins.

**Figure 6:** Performance (ROC) of using enrichment scores of key clusters to classify HCC from ICC: (a) individual ROC curves when using enrichment scores of each cluster separately; (b) combinative ROC curve when using enrichment scores of clusters 1 and 2 together; (c) comparisons of actual enrichment levels of clusters 1 and 2 in two histological groups.

**Figure 7:** The efficacy of the risk model of HCC in predicting survival in TCGA-LIHC. The distribution of risk score and survival status of all samples are shown as (a, b); the heat map of expression of the genes included in the model is shown in (c); (d) Kaplan-Meier plot showing the overall survival based on the relatively high and low risk divided by the optimal cut-off point; (e) time-dependent ROC curve analysis of survival prediction by the prognostic model.

**Figure 8:** The efficacy of the risk model of ICC in predicting survival in TCGA-LIHC. The distribution of risk score and survival status of all samples are shown as (a, b); the heat map of expression of the genes included in the model is shown in (c); (d) Kaplan-Meier plot showing the overall survival based on the relatively high and low risk divided by the optimal cut-off point; (e) time-dependent ROC curve analysis of survival prediction by the prognostic model.

**Figure 9:** Kaplan-Meier plots showing the overall survival based on the relatively high and low risk divided by the optimal cut-off point. Both scoring models were replied to GEO cohorts of HCC (a) and ICC (b). (c) Using the expression level of CYP26A1 to predict overall survival in this ICC cohort; (d) using the expression level of NAT2 to predict overall survival in this ICC cohort.

**Table 1:** Clustering coefficient and enrichment significance of top 9 clusters in PPI network with gene number over or equal to 10.

	Number of nodes	Number of edges	Average node degree	Average local clustering coefficient	Enrichment *p*
*All 217*					
	217	1604	14.8	0.462	<1.0*e* − 16
*Cluster*					
1	22	136	12.4	0.824	<1.0*e* − 16
2	17	78	9.18	0.859	<1.0*e* − 16
3	14	53	7.57	0.795	<1.0*e* − 16
4	13	43	6.62	0.78	<1.0*e* − 16
5	12	39	6.5	0.851	<1.0*e* − 16
6	11	32	5.82	0.78	<1.0*e* − 16
7	11	43	7.82	0.832	<1.0*e* − 16
8	11	47	8.55	0.863	<1.0*e* − 16
9	10	30	6	0.815	<1.0*e* − 16

**Table 2:** The area under curve and confidence intervals when using enrichment scores of each cluster separately to conduct ROC curves.

GSVA score	Area under curve	Confidence intervals
Cluster 1	0.854	0.742-0.966
Cluster 2	0.848	0.737-0.959
Cluster 3	0.584	0.422-0.746
Cluster 4	0.613	0.448-0.777
Cluster 5	0.488	0.321-0.655
Cluster 6	0.728	0.581-0.875
Cluster 7	0.71	0.561-0.859
Cluster 8	0.659	0.497-0.821
Cluster 9	0.584	0.421-0.747

**Table 3:** List of prognostic genes selected from clusters 1 and 2 based on univariate Cox regression analyses.

HCC				
Genes	*p* value	Hazard ratio	Low 95% CI	High 95% CI
*ADH1A*	0.00300914	0.58612961	0.41183469	0.83418889
*ADH1C*	0.01615408	0.65101065	0.45887801	0.92358941
*ADH4*	0.00021488	0.50858731	0.35551424	0.72756874
*ADH6*	0.02940703	0.67874006	0.47891002	0.96195118
*CYP2C8*	0.00763845	0.62287048	0.43988422	0.8819767
*CYP2C9*	0.00178533	0.5729836	0.4040112	0.81262649
*CYP2E1*	0.03361684	0.68402826	0.4818712	0.97099528
*CYP3A4*	0.02265256	0.66736591	0.47133686	0.94492347
*CYP3A43*	0.00376117	0.59530744	0.41915087	0.84549735
*CYP4A11*	0.02017749	0.66161136	0.46692154	0.93747996
*CYP4F2*	0.00494087	0.60667242	0.42816603	0.85959978
*FMO3*	0.00285012	0.58585877	0.41233092	0.83241514
*RDH16*	0.00577881	0.61128672	0.43097773	0.86703195
*RDH5*	0.04857012	0.704856	0.49791407	0.99780667
ICC				
Genes	*p* value	Hazard ratio	Low 95% CI	High 95% CI
*CYP26A1*	0.04156983	0.33466224	0.11678091	0.95905073
*NAT2*	0.02758781	3.25001451	1.13891623	9.2742504
*UGT2B10*	0.0441489	2.92347735	1.02849349	8.30994054

## Data Availability

The datasets generated for this study are available on request to the corresponding authors.

## Supplementary Materials

Supplementary 1 Supplementary Table 1: clinicopathological information of included subjects.

Supplementary 2 Supplementary Table 2: primer sequences for P5 and P7.
